# Inferences for Weibull Fréchet Distribution Using a Bayesian and Non-Bayesian Methods on Gastric Cancer Survival Times

**DOI:** 10.1155/2021/9965856

**Published:** 2021-05-26

**Authors:** Rashad M. EL-Sagheer, Ethar M. Shokr, Mohamed A. W. Mahmoud, Beih S. El-Desouky

**Affiliations:** ^1^Mathematics Department, Faculty of Science, Al-Azhar University, Nasr City, 11884 Cairo, Egypt; ^2^Mathematics Department, Faculty of Science, Mansoura University, Mansoura 35516, Egypt

## Abstract

In this article, based on progressively type-II censored schemes, the maximum likelihood, Bayes, and two parametric bootstrap methods are used for estimating the unknown parameters of the Weibull Fréchet distribution and some lifetime indices as reliability and hazard rate functions. Moreover, approximate confidence intervals and asymptotic variance-covariance matrix have been obtained. Markov chain Monte Carlo technique based on Gibbs sampler within Metropolis–Hasting algorithm is used to generate samples from the posterior density functions. Furthermore, Bayesian estimate is computed under both balanced square error loss and balanced linear exponential loss functions. Simulation results have been implemented to obtain the accuracy of the estimators. Finally, application on the survival times in years of a group of patients given chemotherapy and radiation treatment is presented for illustrating all the inferential procedures developed here.

## 1. Introduction

In recent years, the experiments that it results survival data are less preferred because of being time consuming and expensive. In many situations, use of complete sample is neither possible nor desirable. In such cases, the sample needs to be censored. The value of observation is partially known and incomplete in censoring data. Different types of censoring schemes are interval, type-I, type-II, progressive, hybrid, and random. Among these, type-I and type-II are the two basic censored schemes. In these schemes, the life testing experiment terminates at a prespecified time *T* and number of failures *m*, respectively. For more details and applications, see Lawless [1] and Cohen [2]. The main drawback of them is that it does not apply to all removal points until termination points. For this reason, progressive censoring is proposed. It can be classified into progressive type-I and progressive type-II censoring schemes. In progressive type-I censoring scheme, let *n* be the sample size used in the experiment. In this censoring scheme, *R*_1_, *R*_2_, ⋯, *R*_*m*_ are the number of items which randomly withdrawn at time points *T*_1_, *T*_2_, ⋯, *T*_*m*_, respectively, and the test will be terminated at *T*_*m*_. Now, we describe progressive type-II censoring scheme. Consider *n* units are put on the experiment. We remove randomly *R*_1_ number of survival units when the first failure *Y*_1:*m*:*n*_ is observed. This process continues till the *m*th failure occurs. We assume that the *m*th failure time *Y*_*m*:*m*:*n*_ takes place, and the remaining surviving units is *R*_*m*_ = *n* − *m* − ∑_*k*=1_^*m*−1^*R*_*k*_. So that we assume *R* = (*R*_1_, *R*_2_, ⋯, *R*_*m*_) and *Y* = (*Y*_1:*m*:*n*_, *Y*_2:*m*:*n*_, ⋯, *Y*_*m*:*m*:*n*_), respectively, the censoring scheme and the progressive type-II censored sample. For various applications on this scheme, see [3–8]. The algorithm that used to simulate the sample is discussed in Balakrishnan and Sandhu [9].

The four parameters Weibull Fréchet distribution WFr(*a*, *b*, *α*, *β*) is a generalization of the Weibull and the Fréchet distributions as discussed in Afify et al. [10]. The probability density function (pdf) and cumulative distribution function (cdf) of a random variable *Y* follows WFr(*a*, *b*, *α*, *β*) are given, respectively, by

(1) $$\begin{array}{c} f\left(y\right)=ab\beta \alpha^{\beta }y^{-\beta -1}\exp\left[-b{\left(\frac{\alpha }{y}\right)}^{\beta }\right]\;{\left\{1-\exp\left[-{\left(\frac{\alpha }{y}\right)}^{\beta }\right]\right\}}^{-b-1}\times \exp\left(-a{\left\{\exp\left[{\left(\frac{\alpha }{y}\right)}^{\beta }\right]-1\right\}}^{-b}\right), \end{array}$$

(2) $$\begin{array}{c} F\left(y\right)=1-\exp\left(-a{\left\{\exp\left[{\left(\frac{\alpha }{y}\right)}^{\beta }\right]-1\right\}}^{-b}\right), \end{array}$$

where *a*, *b*, *α*, *β* > 0, *y* > 0, *α* is a scale parameter, and *a*, *b*, and *β* are the shape parameters. Also, the reliability and hazard rate functions of WFr(*a*, *b*, *α*, *β*) are, respectively, given by

(3) $$\begin{array}{c} r\left(t\right)=\exp\left(-a{\left\{\exp\left[{\left(\frac{\alpha }{t}\right)}^{\beta }\right]-1\right\}}^{-b}\right), \end{array}$$

(4) $$\begin{array}{c} h\left(t\right)=ab\beta \alpha^{\beta }t^{-\beta -1}\exp\left(-b{\left(\frac{\alpha }{t}\right)}^{\beta }\right){\left(1-\exp\left[-{\left(\frac{\alpha }{t}\right)}^{\beta }\right]\right)}^{\left(-b-1\right)}. \end{array}$$

The WFr distribution has been shown to be useful for modeling and analyzing the life time data in medical and biological sciences, engineering, etc. So, it has been received the greatest attention from theoretical and applied statisticians primarily due to its use in reliability and life testing studies. This distribution is a very flexible model that approaches to different distributions when its parameters are changed. It contains the following new special models:

1. WFr(*a*, *b*, *α*, 1) follows the Weibull inverse exponential model
2. WFr(*a*, 1, *α*, *β*) is the exponential Fréchet model
3. WFr(*a*, *b*, *α*, 2) refers to the Weibull inverse Rayleigh model
4. WFr(*a*, 1, *α*, 2) reduces to the exponential inverse Rayleigh model
5. WFr(*a*, 1, *α*, 1) follows the exponential inverse exponential model

In this article, the maximum likelihood and Bayesian inference of unknown parameters, as well as reliability and hazard functions, will be studied under progressive type-II censoring scheme. The asymptotic confidence interval of the reliability and hazard functions is approximated by delta method and bootstrap methods. The Markov chain Monte Carlo technique (MCMC) procedure to estimate the parameters and corresponding credible intervals is also discussed which is the great success story of modern day Bayesian statistics. MCMC has a sister method, which is the Gibbs sampling method. They permit the numerical calculation of posterior distributions in situations far too complicated for analytic expression, as demonstrated in Brooks [11]. The specification of the conditional posterior distribution for each parameter only requires for the Gibbs sampler method. In situations where those distributions are simple to sample from, the approach is easily implemented. In other situations, the more complex Metropolis-Hastings approach needs to be considered, see Gupta et al. [12]. Moreover, all results of this paper were made using the Mathematica version 12 software.

The remainder of this article is organized as follows: In Section 2, the MLEs for the unknown parameters, reliability, and hazard rate functions are estimated. Asymptotic confidence intervals (ACIs) based on MLEs are discussed in Section 3. In Section 4, two parametric bootstrap CIs are constructed.  Section 5 provides the conditional distributions required for implementing the Markov chain Monte Carlo to derive the Bayes estimates with respect to two loss functions (BSE and BLINEX). Two examples, one of them used simulated data and the other used a real data sets, have been analyzed in Section 6. Eventually, conclusion is inserted in Section 7.

## 2. ML Inference

Let $\underline{y}=Y_{1:m:n},Y_{2:m:n},\cdots ,Y_{m:m:n}$ be a prog. type-II censored sample from WFD with the censored scheme (*R*_1_, *R*_2_, ⋯, *R*_*m*_). From Eqs. (1) and (2), the log-likelihood function $\ell =\ln\left(L\left(a,b,\alpha ,\beta |\underline{y}\right)\right)$ is:

(5) $$\begin{array}{c} \ell \propto m\;\ln\left(a\right)+m\;\ln\left(b\right)+m\;\ln\left(\beta \right)+m\beta \;\ln\left(\alpha \right)-\left(\beta +1\right)\overset{m}{\underset{k=1}{\sum }}\ln\left(y_{k}\right)-b\overset{m}{\underset{k=1}{\sum }}{\left(\frac{\alpha }{y_{k}}\right)}^{\beta }-a\overset{m}{\underset{k=1}{\sum }}\left(R_{k}+1\right){\left(\exp\left[{\left(\frac{\alpha }{y_{k}}\right)}^{\beta }\right]-1\right)}^{-b}-\left(b+1\right)\overset{m}{\underset{k=1}{\sum }}\ln\left[1-\exp\left[-{\left(\frac{\alpha }{y_{k}}\right)}^{\beta }\right]\right]. \end{array}$$

Then, the normal equations to obtain estimates of unknown parameters are given by:

(6) $$\begin{array}{c} \frac{m}{a}-\overset{m}{\underset{k=1}{\sum }}\left(R_{k}+1\right){\left(\exp\left[{\left(\frac{\alpha }{y_{k}}\right)}^{\beta }\right]-1\right)}^{-b}=0, \end{array}$$

(7) $$\begin{array}{c} \frac{m}{b}-\overset{m}{\underset{k=1}{\sum }}{\left(\frac{\alpha }{y_{k}}\right)}^{\beta }+a\overset{m}{\underset{k=1}{\sum }}\left(R_{k}+1\right){\left(\exp\left[{\left(\frac{\alpha }{y_{k}}\right)}^{\beta }\right]-1\right)}^{-b}\ln\left(\exp\left[{\left(\frac{\alpha }{y_{k}}\right)}^{-b}\right]-1\right)-\overset{m}{\underset{k=1}{\sum }}\ln\left(1-\exp\left[-{\left(\frac{\alpha }{y_{k}}\right)}^{\beta }\right]\right)=0, \end{array}$$

(8) $$\begin{array}{c} \frac{m\beta }{\alpha }-b\overset{m}{\underset{k=1}{\sum }}\left(\frac{\beta }{y_{k}}\right){\left(\frac{\alpha }{y_{k}}\right)}^{\beta -1}-\left(1+b\right)\overset{m}{\underset{k=1}{\sum }}\frac{\beta {\left(\alpha /y_{k}\right)}^{\beta -1}\exp\left[-{\left(\alpha /y_{k}\right)}^{\beta }\right]}{\left(1-\exp\left[-{\left(\alpha /y_{k}\right)}^{\beta }\right]\right)\times y_{k}}+ab\beta \overset{m}{\underset{k=1}{\sum }}\left(R_{k}+1\right){\left(\frac{\alpha }{y_{k}}\right)}^{\beta -1}\exp\left[{\left(\frac{\alpha }{y_{k}}\right)}^{\beta }\right]{\left(\exp\left[{\left(\frac{\alpha }{y_{k}}\right)}^{\beta }\right]-1\right)}^{-b-1}\frac{1}{y_{k}}=0, \end{array}$$

(9) $$\begin{array}{c} \frac{m}{\beta }+m\;\ln\left(\alpha \right)-\overset{m}{\underset{k=1}{\sum }}\ln\left(y_{k}\right)-b\overset{m}{\underset{k=1}{\sum }}{\left(\frac{\alpha }{y_{k}}\right)}^{\beta }\ln\left(\frac{\alpha }{y_{k}}\right)-\left(1+b\right)\overset{m}{\underset{k=1}{\sum }}\frac{{\left(\alpha /y_{k}\right)}^{\beta }\exp\left[-{\left(\alpha /y_{k}\right)}^{\beta }\right]\ln\left(\alpha /y_{k}\right)}{1-\exp\left[-{\left(\alpha /y_{k}\right)}^{\beta }\right]}+ab\overset{m}{\underset{k=1}{\sum }}\left(R_{k}+1\right)\ln\left(\frac{\alpha }{y_{k}}\right)\exp\left[{\left(\frac{\alpha }{y_{k}}\right)}^{\beta }\right]{\left(\exp\left[{\left(\frac{\alpha }{y_{k}}\right)}^{\beta }\right]-1\right)}^{-b-1}{\left(\frac{\alpha }{y_{k}}\right)}^{\beta }=0. \end{array}$$

Hence, from Eq. (6), we get

(10) $$\begin{array}{c} \hat{a}=m{\left[\overset{m}{\underset{k=1}{\sum }}\left(R_{k}+1\right){\left(\exp\left[{\left(\frac{\alpha }{y_{k}}\right)}^{\beta }\right]-1\right)}^{-b}\right]}^{-1}. \end{array}$$

By using Newton-Raphson iteration method to solve Eqs. (7)–(10), we get the MLEs of the unknown parameters $\hat{a},\hat{b},\hat{\alpha }$, and $\hat{\beta }$. Moreover, $\hat{r}\left(t\right)$ and $\hat{h}\left(t\right)$ are obtained by replacing *a*, *b*, *α*, and *β* with $\hat{a},\hat{b},\hat{\alpha }$, and $\hat{\beta }$ in Eqs. (3) and (4). For more details, see EL-Sagheer [3].

## 3. Approximate Confidence Intervals

This section, to obtain 100(1 − *δ*) CI for the parameters using asymptotic Fisher information matrix $\hat{I}\left(a,b,\alpha ,\beta \right)$ which is given by

(11) $$\begin{array}{c} \hat{I}\left(a,b,\alpha ,\beta \right)={\left(\begin{array}{cccc} -\frac{\partial^{2}\ell }{\partial a^{2}} & -\frac{\partial^{2}\ell }{\partial a\partial b} & -\frac{\partial^{2}\ell }{\partial a\partial \alpha } & -\frac{\partial^{2}\ell }{\partial a\partial \beta }\\ -\frac{\partial^{2}\ell }{\partial b\partial a} & -\frac{\partial^{2}\ell }{\partial b^{2}} & -\frac{\partial^{2}\ell }{\partial b\partial \alpha } & -\frac{\partial^{2}\ell }{\partial b\partial \beta }\\ -\frac{\partial^{2}\ell }{\partial \alpha \partial a} & -\frac{\partial^{2}\ell }{\partial \alpha \partial b} & -\frac{\partial^{2}\ell }{\partial \alpha^{2}} & -\frac{\partial^{2}\ell }{\partial \alpha \partial \beta }\\ -\frac{\partial^{2}\ell }{\partial \beta \partial a} & -\frac{\partial^{2}\ell }{\partial \beta \partial b} & -\frac{\partial^{2}\ell }{\partial \beta \partial \alpha } & -\frac{\partial^{2}\ell }{\partial \beta^{2}} \end{array}\right)}_{↓\left\{a=\hat{a},b=\hat{b},\alpha =\hat{\alpha },\beta =\hat{\beta }\right\}}. \end{array}$$

Therefore, the asymptotic variance-covariance matrix is given by

(12) $$\begin{array}{c} \hat{V}={\overset{\wedge }{I}}^{-1}\left(\hat{a},\hat{b},\hat{\alpha },\hat{\beta }\right)={\left(\begin{array}{cccc} \hat{\mathrm{var}\left(a\right)} & \hat{\mathrm{cov}\left(a,b\right)} & \hat{\mathrm{cov}\left(a,\alpha \right)} & \hat{\mathrm{cov}\left(a,\beta \right)}\\ \hat{\mathrm{cov}\left(b,a\right)} & \hat{\mathrm{var}\left(b\right)} & \hat{\mathrm{cov}\left(b,\alpha \right)} & \hat{\mathrm{cov}\left(b,\beta \right)}\\ \hat{\mathrm{cov}\left(\alpha ,a\right)} & \hat{\mathrm{cov}\left(\alpha ,b\right)} & \hat{\mathrm{var}\left(\alpha \right)} & \hat{\mathrm{cov}\left(\alpha ,\beta \right)}\\ \hat{\mathrm{cov}\left(\beta ,a\right)} & \hat{\mathrm{cov}\left(\beta ,b\right)} & \hat{\mathrm{cov}\left(\beta ,\alpha \right)} & \hat{\mathrm{var}\left(\beta \right)} \end{array}\right)}_{↓\left\{\hat{a},\hat{b},\hat{\alpha },\hat{\beta }\right\}}. \end{array}$$

Hence, *a*, *b*, *α*, and *β* are approximately normal distribution with mean vector $\left(\hat{a},\hat{b},\hat{\alpha },\hat{\beta }\right)$ and covariance matrix ${\overset{\wedge }{I}}^{-1}\left(a,b,\alpha ,\beta \right)$. Thus, the (1 − *δ*)100% ACIs for *a*, *b*, *α*, and *β* are given by

(13) $$\begin{array}{c} \left[\hat{a}\pm Z_{\delta /2}\sqrt{\hat{\mathrm{var}\left(a\right)}}\right],\\ \left[\hat{b}\pm Z_{\delta /2}\sqrt{\hat{\mathrm{var}\left(b\right)}}\right],\\ \left[\hat{\alpha }\pm Z_{\delta /2}\sqrt{\hat{\mathrm{var}\left(\alpha \right)}}\right],\\ \left[\hat{\beta }\pm Z_{\delta /2}\sqrt{\hat{\mathrm{var}\left(\beta \right)}}\right], \end{array}$$

where *Z*_*δ*/2_ is the percentile of the standard normal distribution with right-tail probability *δ*/2. Further, the asymptotic confidence intervals for *r*(*t*) and *h*(*t*) are obtained by using delta method (see Greene [13]). Let *B*′_1_ = (*∂r*(*t*)/*∂a*, *∂r*(*t*)/*∂b*, *∂r*(*t*)/*∂α*, *∂r*(*t*)/*∂β*) and $B\prime_{2}=\left(\begin{array}{cccc} \partial h\left(t\right)/\partial a, & \partial h\left(t\right)/\partial b, & \partial h\left(t\right)/\partial \alpha , & \partial h\left(t\right)/\partial \beta \end{array}\right)$. Thus, the variances of $\hat{r}\left(t\right)$ and $\hat{h}\left(t\right)$ are given by

(14) $$\begin{array}{c} \hat{\mathrm{var}}\left(\hat{r}\left(t\right)\right)≃{\left[B_{1}^{\prime }{\overset{\wedge }{I}}^{-1}B_{1}\right]}_{↓\left\{\hat{a},\hat{b},\hat{\alpha },\hat{\beta }\right\}},\\ \hat{\mathrm{var}}\left(\hat{h}\right)≃{\left[B_{2}^{\prime }{\overset{\wedge }{I}}^{-1}B_{2}\right]}_{↓\left\{\hat{a},\hat{b},\hat{\alpha },\hat{\beta }\right\}}. \end{array}$$

Thus, the (1 − *δ*)100% ACIs for *r*(*t*) and *h*(*t*) are

(15) $$\begin{array}{c} \left[\hat{r}\pm Z_{\delta /2}\sqrt{\hat{\mathrm{var}\left(r\right)}}\;\right],\\ \left[\hat{h}\pm Z_{\delta /2}\sqrt{\hat{\mathrm{var}\left(h\right)}}\;\right]. \end{array}$$

## 4. Bootstrap Confidence Intervals

It is seen in the previous section that second order derivatives are required to obtain ACIs of the unknown model parameters, which is cumbersome. So, we consider bootstrap technique. In particular, we adopt percentile bootstrap (Boot-p) (see Efron [14]) and bootstrap-t (Boot-t) (see Hall [15]) techniques.

### 4.1. Parametric Boot-p CI

Here, we describe the algorithm how to obtain the confidence intervals using Boot-p method. First, we obtain the MLEs of *ψ* = (*a*, *b*, *α*, *β*, *r*(*t*), *h*(*t*)) by solving Eqs. (7)–(10) and denoted them by $\hat{\psi }=\left(\hat{a},\hat{b},\hat{\alpha },\hat{\beta },\hat{r}\left(t\right),\hat{h}\left(t\right)\right)$; then, the bootstrap sample *x*^∗^ = (*x*_1_^∗^, *x*_2_^∗^, ⋯, *x*_*m*_^∗^) has to be generated. We compute ${\overset{\wedge }{\psi }}^{*}=\left({\overset{\wedge }{a}}^{*},{\overset{\wedge }{b}}^{*},{\overset{\wedge }{\alpha }}^{*},{\overset{\wedge }{\beta }}^{*},{\overset{\wedge }{r}}^{*}\left(t\right),{\overset{\wedge }{h}}^{*}\left(t\right)\right)$ based on *x*^∗^. Repeat this procedure for *N*boot times to get ${\hat{\psi }}_{1}^{*},{\hat{\psi }}_{2}^{*},\cdots ,{\hat{\psi }}_{N\text{boot}}^{*}$, where ${\hat{\psi }}_{i}^{*}=\left({\hat{a}}_{i}^{*},{\hat{b}}_{i}^{*},{\hat{\alpha }}_{i}^{*},{\hat{\beta }}_{i}^{*},{\hat{r}}_{i}^{*}\left(t\right),{\hat{h}}_{i}^{*}\left(t\right)\right)$, *i* = 1, 2, ⋯, *N*boot. Next, we arrange ${\hat{\psi }}_{i}^{*}$ in ascending order and denote them by ${\hat{\psi }}_{\left(1\right)}^{*},{\hat{\psi }}_{\left(2\right)}^{*},\cdots ,{\hat{\psi }}_{\left(N\text{boot}\right)}^{*}$. Thus, the (1 − *δ*)100% approximate bootstrap-p confidence interval for *ψ* is obtained as (*L*, *U*), where $L={\hat{\psi }}_{Nboot\left(\delta /2\right)}^{*}$ and $U={\hat{\psi }}_{N\text{boot}\left(1-\left(\delta /2\right)\right)}^{*}$.

### 4.2. Parametric Boot-t CI

The Boot-p method does not perform well when sample size is small. So, in this subsection, we discuss the Boot-t method, which is simple to apply compared with Boot-p method. We obtain ${\overset{\wedge }{\psi }}^{*}=\left({\overset{\wedge }{a}}^{*},{\overset{\wedge }{b}}^{*},{\overset{\wedge }{\alpha }}^{*},{\overset{\wedge }{\beta }}^{*},{\overset{\wedge }{r}}^{*}\left(t\right),{\overset{\wedge }{h}}^{*}\left(t\right)\right)$ similar to the procedure as mentioned in Boot-p method. Then, based on the bootstrap sample *x*^∗^ = *x*_1_^∗^, *x*_2_^∗^, ⋯, *x*_*m*_^∗^, we compute the variance-covariance matrix ${\hat{I}}_{x^{*}}^{-1}\left({\overset{\wedge }{a}}^{*},{\overset{\wedge }{b}}^{*},{\overset{\wedge }{\alpha }}^{*},{\overset{\wedge }{\beta }}^{*}\right)$. For *i* = 1, 2, ⋯, *N*boot calculate the value of the statistic $T_{\psi_{i}}^{*}=\left({\hat{\psi }}_{i}^{*}-{\hat{\psi }}_{i}\right)/\sqrt{\hat{\mathrm{var}\left(\psi_{i}^{*}\right)}}$. Then, we arrange them in ascending order and get *T*_*ψ*_(1)__^∗^, *T*_*ψ*_(2)__^∗^, ⋯, *T*_*ψ*_(*N*boot)__^∗^. Thus, the (1 − *δ*)100% approximate bootstrap-t confidence interval for *ψ* is obtained as (*L*, *U*), where $L={\hat{\psi }}_{i}+\sqrt{\hat{\mathrm{var}\left(\psi_{i}^{*}\right)}}*T_{\psi_{\left(N\text{boot}\left(\delta /2\right)\right)}}^{*}$ and $U={\hat{\psi }}_{i}+\sqrt{\hat{\mathrm{var}\left(\psi_{i}^{*}\right)}}*T_{\psi_{\left(N\text{boot}\left(1-\left(\delta /2\right)\right)\right)}}^{*}$.

## 5. Bayesian Inference

In this section, we obtain Bayes estimates and the corresponding credible intervals for the parameters *a*, *b*, *α*, and *β* and the reliability characteristics functions *r*(*t*) and *h*(*t*). To do this, we let the prior distributions for them are independent Gamma distributions with different and known hyperparameters, i.e., *a* ~ Gamma(*c*1, *k*1), *b* ~ Gamma(*c*2, *k*2), *α* ~ Gamma(*c*3, *k*3), and *β* ~ Gamma(*c*4, *k*4), where *c*_1_, *k*_1_, *c*_2_, *k*_2_, *c*_3_, *k*_3_, *c*_4_, *k*_4_ > 0. Hence, the posterior distribution of *a*, *b*, *α*,and *β* given sample vector $\underline{y}$ is

(16) $$\begin{array}{c} \pi^{*}\left(a,b,\alpha ,\beta \;|\;\underline{y}\right)\propto a^{m+c_{1}-1}b^{m+c_{2}-1}\alpha^{m\beta +c_{3}-1}\beta^{m+c_{4}-1}\overset{m}{\underset{k=1}{\prod }}{\left(y_{k}\right)}^{-\beta -1}\overset{m}{\underset{k=1}{\prod }}{\left(1-\exp\left[-{\left(\frac{\alpha }{y_{k}}\right)}^{\beta }\right]\right)}^{-b-1}\times \exp\left[\overset{m}{\underset{k=1}{\sum }}-b{\left(\frac{\alpha }{y_{k}}\right)}^{\beta }-a\overset{m}{\underset{k=1}{\sum }}\left(R_{k}+1\right){\left(\exp\left[{\left(\frac{\alpha }{y_{k}}\right)}^{\beta }\right]-1\right)}^{-b}-k_{1}a-k_{2}b-k_{3}\alpha -k_{4}\beta \right]. \end{array}$$

Hence, the conditional posterior densities of *a*, *b*, *α*, and *β* are as follows:

(17) $$\begin{array}{c} \pi_{1}^{*}\left(a\;|\;b,\alpha ,\beta ,\underline{y}\right)\propto a^{m+c_{1}-1}\exp\left[-a\overset{m}{\underset{k=1}{\sum }}\left(R_{k}+1\right){\left(\exp\left[{\left(\frac{\alpha }{y_{k}}\right)}^{\beta }\right]-1\right)}^{-b}-k_{1}a\right], \end{array}$$

(18) $$\begin{array}{c} \pi_{2}^{*}\left(b\;|\;a,\alpha ,\beta ,\underline{y}\right)\propto b^{m+c_{2}-1}\overset{m}{\underset{k=1}{\prod }}{\left(1-\exp\left[-{\left(\frac{\alpha }{y_{k}}\right)}^{\beta }\right]\right)}^{-b-1}\times \exp\left[\overset{m}{\underset{k=1}{\sum }}-b{\left(\frac{\alpha }{y_{k}}\right)}^{\beta }-a\overset{m}{\underset{k=1}{\sum }}\left(R_{k}+1\right){\left(\exp\left[{\left(\frac{\alpha }{y_{k}}\right)}^{\beta }\right]-1\right)}^{-b}-k_{2}b\right], \end{array}$$

(19) $$\begin{array}{c} \pi_{3}^{*}\left(\alpha \;|\;a,b,\beta ,\underline{y}\right)\propto \alpha^{m\beta +c_{3}-1}\overset{m}{\underset{k=1}{\prod }}{\left(1-\exp\left[-{\left(\frac{\alpha }{y_{k}}\right)}^{\beta }\right]\right)}^{-b-1}\times \exp\left[\overset{m}{\underset{k=1}{\sum }}-b{\left(\frac{\alpha }{y_{k}}\right)}^{\beta }-a\overset{m}{\underset{k=1}{\sum }}\left(R_{k}+1\right){\left(\exp\left[{\left(\frac{\alpha }{y_{k}}\right)}^{\beta }\right]-1\right)}^{-b}-k_{3}\alpha \right], \end{array}$$

(20) $$\begin{array}{c} \pi_{4}^{*}\left(\beta \;|\;a,b,\alpha ,\underline{y}\right)\propto \beta^{m+c_{4}-1}\overset{m}{\underset{k=1}{\prod }}{\left(y_{k}\right)}^{-\beta -1}\overset{m}{\underset{k=1}{\prod }}{\left(1-\exp\left[-{\left(\frac{\alpha }{y_{k}}\right)}^{\beta }\right]\right)}^{-b-1}\times \exp\left[\overset{m}{\underset{k=1}{\sum }}-b{\left(\frac{\alpha }{y_{k}}\right)}^{\beta }-a\overset{m}{\underset{k=1}{\sum }}\left(R_{k}+1\right){\left(\exp\left[{\left(\frac{\alpha }{y_{k}}\right)}^{\beta }\right]-1\right)}^{-b}-k_{4}\beta \right]. \end{array}$$

From Eq. (17), the full conditional posterior density of *a* is Gamma(*m* + *c*_1_, *k*_1_ + ∑_*i*=1_^*m*^(*R*_*i*_ + 1)(exp[(*α*/*x*_*i*_)^*β*^] − 1)^−*b*^). Thus, the samples of *a* can be generated by using any gamma routine. From Eqs. (18), (19), and (20), the posterior of *b*, *α*, and *β* do not present standard form, but the plots of them show that they are similar to normal distribution, see Figures 1–3, i.e., all the conditional posterior distributions contain a single maximum value, and this allows us to apply MCMC. Therefore, we generate random samples from these distributions using the Metropolis-Hastings algorithm with the normal proposal distribution, see Tierney [16]. The Metropolis–Hastings algorithm within Gibbs sampling:

(1) Start with (*a*^(0)^, *b*^(0)^, *α*^(0)^, *β*^(0)^)
(2) Set *k* = 1
(3) Generate *a*^(*k*)^ from Gamma(*m* + *c*_1_, *k*_1_ + ∑_*j*=1_^*m*^(*R*_*j*_ + 1)(exp[(*α*^(*k* − 1)^/*y*_*j*_)^*β*^(*k* − 1)^^] − 1)^−*b*^(*k* − 1)^^)
(4) Using M-H
  - Generate *b*^∗^ from *N*(*b*^(*k* − 1)^, var(*b*)), *α*^∗^ from *N*(*α*^(*k* − 1)^, var(*α*)), and *β*^∗^ from *N*(*β*^(*k* − 1)^, var(*β*))
  - Evaluate the acceptance probabilities

(21) $$\begin{array}{c} \psi_{1}=\min\left[1,\frac{\pi_{2}^{*}\left(b^{*}\;|\;a^{\left(k\right)},\alpha^{\left(k-1\right)},\beta^{\left(k-1\right)},\underline{y}\right)}{\pi_{2}^{*}\left(b^{\left(k-1\right)}\;|\;a^{\left(k\right)},\alpha^{\left(k-1\right)},\beta^{\left(k-1\right)},\underline{y}\right)}\right],\\ \psi_{2}=\min\left[1,\frac{\pi_{3}^{*}\left(\alpha^{*}\;|\;a^{\left(k\right)},b^{\left(k\right)},\beta^{\left(k-1\right)},\underline{y}\right)}{\pi_{3}^{*}\left(\alpha^{\left(k-1\right)}\;|\;a^{\left(k\right)},b^{\left(k\right)},\beta^{\left(k-1\right)},\underline{y}\right)}\right],\\ \psi_{3}=\min\left[1,\frac{\pi_{4}^{*}\left(\beta^{*}\;|\;a^{\left(k\right)},b^{\left(k\right)},\alpha^{\left(k\right)},\underline{y}\right)}{\pi_{4}^{*}\left(\beta^{\left(k-1\right)}\;|\;a^{\left(k\right)},b^{\left(k\right)},\alpha^{\left(k\right)},\underline{y}\right)}\right], \end{array}$$

(c) Generate *r*1, *r*2, and *r*3 from a Uniform(0, 1) distribution
(d) If *r*1 < *ψ*_1_, accept the proposal, and set *b*^(*k*)^ = *b*^∗^; else, set *b*^(*k*)^ = *b*^(*k* − 1)^
(e) If *r*2 < *ψ*_2_, set *α*^(*k*)^ = *α*^∗^; otherwise, set *α*^(*k*)^ = *α*^(*k* − 1)^
(f) If *r*3 < *ψ*_3_, set *β*^(*k*)^ = *β*^∗^; otherwise, set *β*^(*k*)^ = *β*^(*k* − 1)^

(5) Evaluate the reliability characteristics *r*(*t*) and *h*(*t*)

(22) $$\begin{array}{c} r^{\left(k\right)}\left(t\right)=\exp\left(-a^{\left(k\right)}{\left\{\exp\left[{\left(\frac{\alpha^{\left(k\right)}}{t}\right)}^{\beta^{\left(k\right)}}\right]-1\right\}}^{-b^{\left(k\right)}}\right),\\ h^{\left(k\right)}\left(t\right)=a^{\left(k\right)}b^{\left(k\right)}\beta^{\left(k\right)}{\left(\alpha^{\left(k\right)}\right)}^{\beta^{\left(k\right)}}t^{-\beta^{\left(k\right)}-1}\exp\left(-b^{\left(k\right)}{\left(\frac{\alpha^{\left(k\right)}}{t}\right)}^{\beta^{\left(k\right)}}\right)\times {\left(1-\exp\left[-{\left(\frac{\alpha^{\left(k\right)}}{t}\right)}^{\beta^{\left(k\right)}}\right]\right)}^{\left(-b^{\left(k\right)}-1\right)}. \end{array}$$

(6) Set *k* = *k* + 1
(7) Repeat Steps 3-6 *N* times

Hence, to guarantee the convergence and to remove the affection of the selection of initial value, we remove the first *M* simulated values. Then, the selected samples are *a*^(*k*)^, *b*^(*k*)^, *α*^(*k*)^, *α*^(*k*)^, *β*^(*k*)^, *r*^(*k*)^(*t*), and *h*^(*k*)^(*t*), *k* = *M* + 1, ⋯, *N*; for large *N*, the Bayes estimate of *ν* = *a*, *b*, *α*, *β*, *r*(*t*), or *h*(*t*) is given by

(23) $$\begin{array}{c} {\hat{\nu }}_{MC}=\frac{1}{N-M}\overset{N}{\underset{k=M+1}{\sum }}\nu^{\left(k\right)}. \end{array}$$

To compute the credible intervals of *a*, *b*, *α*, *β*, *r*(*t*), and *h*(*t*), make *a*^(*k*)^, *b*^(*k*)^, *α*^(*k*)^, *β*^(*k*)^, *r*^(*k*)^(*t*), and *h*^(*k*)^(*t*), *k* = 1, 2, ⋯, *N* in ascending order as {*a*^(1)^<⋯<*a*^(*N*)^}, {*b*^(1)^<⋯<*b*^(*N*)^}, {*α*^(1)^<⋯<*α*^(*N*)^}, {*β*^(1)^<⋯<*β*^(*N*)^}, {*r*^(1)^(*t*)<⋯<*r*^(*N*)^(*t*)}, and {*h*^(1)^(*t*)<⋯<*h*^(*N*)^(*t*)}; hence, (1 − *δ*)100% CI of *a*, *b*, *α*, *β*, *r*(*t*), or *h*(*t*) is given by

(24) $$\begin{array}{c} \left[\nu_{\left(N\left(\delta /2\right)\right)},\nu_{\left(N\left(1-\left(\delta /2\right)\right)\right)}\right]. \end{array}$$

### 5.1. Balanced Loss Functions

In this subsection, two loss functions have been considered: (i) balanced squared error loss function and (ii) balanced-LINEX loss function are introduced by Jozani et al. [17]. Let *δ* be an estimator of the unknown parameter *ψ*.  Table 1 represents Bayes estimates of *ψ* under BSE and BLINEX loss functions, where *w* and *q* are both nonzero real numbers.

## 6. Simulation Results and Real Data Analysis

To compare the parameter estimators, we perform Monte Carlo simulations 1000 prog. type-II censored samples for each simulations. MATHEMATICA ver. 12 has been used for all computations, with parameters *a* = 0.5, *b* = 0.5, *α* = 2.0, and *β* = 3.5. The true values of *r*(*t*) and *h*(*t*) at *t* = 0.5 are *r*(0.5) = 0.9879 and *h*(0.5) = 0.1. We also computed the Bayes estimates based on 10000 MCMC samples with respect to the BSE and BLINEX loss function are computed for two distinct values of *ω*, equal 0 and 0.6.

We use the following scheme (CS)in our study:

(25) $$\begin{array}{c} \begin{array}{ccc} \text{CS I} & R_{1}=n-m & R_{i}=0\text{ for }i\neq 1,\\ \text{CS II} & R_{\left(m+1\right)/2}=n-m & R_{i}=0\text{ for }i\neq \frac{\left(m+1\right)}{2}\text{ if }m\text{ odd},\\ & R_{m/2}=n-m & R_{i}=0\text{ for }i\neq \frac{m}{2}\text{ if }m\text{ even},\\ \text{CS III} & R_{m}=n-m & R_{i}=0\text{ for }i\neq \text{m}. \end{array} \end{array}$$

The performance of the resulting estimators of *a*, *b*, *α*, *β*, *r*(*t*), and *h*(*t*) has been considered in terms of mean square error (MSE), which is computed by $MSE=1/M\sum_{i=1}^{M}{\left({\overset{\wedge }{\psi }}_{k}^{i}-\psi_{k}\right)}^{2}$, *k* = 1, 2, ⋯, 6 and *ψ*_1_ = *a*, *ψ*_2_ = *b*, *ψ*_3_ = *α*, *ψ*_4_ = *β*, *ψ*_5_ = *r*(*t*), and *ψ*_6_ = *h*(*t*). All results are shown in Tables 2–7.

### 6.1. Simulated Data Set

In this subsection, we present a simulation example to check the estimation procedures. By using the algorithm described in Balakrishnan and Sandhu [9], we generate sample from WFD(*a*, *b*, *α*, *β*) with the parameters (*a* = .5, *b* = 2.5, *α* = .96, *β* = .6), using progressive censoring scheme CS: *m* = 15 which generated randomly of sample size *n* = 30 with censoring scheme *R* = 7, 1, 2, 4, 1, 0, 0, 0, 0, 0, 0, 0, 0, 0, 0. The progressive type-II censored sample is

(26) $$\begin{array}{c} \begin{array}{cccccccc} 0.2332 & 0.3186 & 0.7247 & 0.854 & 1.0203 & 1.0555 & 1.3103 & 1.3759\\ 1.4376 & 1.4585 & 1.61 & 1.7332 & 1.9045 & 2.1138 & 2.987 & \end{array}. \end{array}$$

From Eqs. (3) and (4), the actual values of *r*(*t*) and *h*(*t*) are 0.9435 and 0.3013, respectively, for *t* = 0.5.

1. Table 8 describes the point estimation for the parameters *a*, *b*, *α*, *β*, *r*(*t*), and *h*(*t*) using MLE, Bootstrap-p, Bootstrap-t, and MCMC methods
2. Table 9 describes 95% CIs for *a*, *b*, *α*, *β*, *r*(*t*), and *h*(*t*) using MLE, Bootstrap-p, Bootstrap-t, and MCMC methods
3. Table 10 describes MCMC results{Mean, Median, Mood, Variance, Standard Deviation, Skewness} for *a*, *b*, *α*, *β*, *r*(*t*), and *h*(*t*)
4. Table 11 describes the Bayesian estimation results under both BSEL and BLINEX with *q* = −0.5,0, 0.5 shape parameter of LINEX loss function and various values of *ω* = 0,0.3,0.6,0.9 for unknown parameters *a*, *b*, *α*, *β*, *r*(*t*), and *h*(*t*)

### 6.2. Survival Times Application

In this subsection, we study an application of a real data set. This data set represents the life data regarding gastric cancer survival times in years for a group of patients given chemotherapy and radiation treatment. This data set reported by Stablein et al. [18] and used in EL-Sagheer and Ahsanullah [19] and Bekker et al. [20]. The data consisting of 46 survival times for 46 patients are:

(27) $$\begin{array}{c} \begin{array}{cccccccccc} 0.047 & 0.115 & 0.121 & 0.132 & 0.164 & 0.197 & 0.203 & 0.260 & 0.282 & 0.296\\ 0.334 & 0.395 & 0.458 & 0.466 & 0.501 & 0.507 & 0.529 & 0.534 & 0.540 & 0.570\\ 0.641 & 0.644 & 0.696 & 0.841 & 0.863 & 1.099 & 1.219 & 1.271 & 1.326 & 1.447\\ 1.485 & 1.553 & 1.581 & 1.589 & 2.178 & 2.343 & 2.416 & 2.444 & 2.825 & 2.830\\ 3.578 & 3.658 & 3.743 & 3.978 & 4.003 & 4.033 & & & & \end{array}, \end{array}$$

for the purpose of the goodness of fit test, the Kolmogorov–Smirnov (KS) distance between the empirical and the fitted distribution functions have been computed. It is 0.0892, and the associated *p* value is 0.826301. Hence, *p* value is quite large; we accept the null hypothesis that the data is coming from the WFr distribution.  Figure 4 describes the empirical and the pdf of WFr, and it shows that the WFr distribution fits the data very well. Now, let we consider progressive type-II censored sample with total sample size *n* = 46, the failure sample size *m* = 26, by using the algorithm described in Balakrishnan and Sandhu [9] with censoring scheme with binomial removal (*p* = 0.4) *R* = {7, 7, 1, 1, 1, 0, 1, 2, 0, 0, 0, 0, 0, 0, 0, 0, 0, 0, 0, 0, 0, 0, 0, 0, 0, 0}. Based on these data, we compute the proposed estimates for the unknown parameters, reliability, and hazard rate functions by various methods (MLEs, Boot-p, Boot-t confidence intervals, and Bayesian estimation).

1. Table 12 describes the point estimation using MLE, Bootstrap-p, Bootstrap-t CI, and MCMC methods

(2) Table 13 describes 95% CI for unknown parameter, reliability, and hazard rate functions using MLE, Bootstrap-p, Bootstrap-t, and MCMC methods

(3) Table 14 describes MCMC results{Mean, Median, Mood, Variance, Standard Deviation, Skewness} for *a*, *b*, *α*, *β*, *r*(*t*), and *h*(*t*)

(4) Table 15 describes a comparison between the results MLE and Bayesian estimation under BSEL and BLINEX loss function

## 7. Conclusion

In this paper, we estimated the parameters, reliability, and hazard rate function of the Weibull Fréchet distribution under progressive type-II censored sample using several methods as MLE, parametric bootstrap, and Bayes estimate. Furthermore, the approximately confidence intervals for these parameters were constructed by using the asymptotic normality of MLE as well as the delta method is used to construct the CIs for the reliability and hazard functions, parametric bootstrap, and Bayes methods. It is clear that the Bayes estimators cannot be obtained in explicit forms, and they can be obtained by using the numerical integration. Because of that, MCMC techniques have been used, and it is observed that the Bayes estimate with respect to informative prior works quite well in this case. Also, the Bayes estimates have been computed with respect to two loss functions. Also, we considered a real life data set for illustrative purpose. Finally, an elaborate simulation study was conducted for different sample sizes (*n*, *m*) and different CSs (I, II, III) for the comparison of the proposed estimates. From the results, we observe the following:

1. Tables 2–7 show that the MSEs decrease as the sample size increases, and Bayesian estimates have the smallest MSEs for *a*, *b*, *α*, *β*, *r*(*t*), and *h*(*t*). So, Bayes estimates perform better than the MLEs and bootstrap methods in all cases considered
2. It is clear that the bootstrap-t is better than MLE and bootstrap-p from (2–7)
3. When *ω* = 0, Bayes estimates are giving better estimates for the unknown parameters and the reliability characteristics in the sense of having smaller MSEs
4. Bayes estimation under BLINEX with *q* = 0.5 provides better estimation in the sense of having smaller MSEs when *ω* = 0 and 0.6
5. For the same sample size, SC I performs better than SC II and SC III in the sense of having smaller MSEs

## Figures and Tables

**Figure 1:** Posterior density function $\pi_{2}^{*}\left(b|a,\alpha ,\beta ,\underline{y}\right)$ of *b*.

**Figure 2:** Posterior density function $\pi_{3}^{*}\left(\alpha |a,b,\beta ,\underline{y}\right)$ of *α*.

**Figure 3:** Posterior density function $\pi_{4}^{*}\left(\beta |a,b,\alpha ,\underline{y}\right)$ of *β*.

**Figure 4:** Fitness of real data.

**Table 1:** Loss functions and the corresponding form of the Bayes estimates.

Loss function name	Loss function Eq.	Bayes estimations
BSEL	$\delta_{w}\left(\underline{x}\right)=w\delta_{0}\left(\underline{x}\right)+\left(1-w\right)E\left(\psi |\underline{x}\right)$	$w\hat{\psi }+\frac{1-w}{N-M}\overset{N}{\underset{i=M}{\sum }}\psi^{\left(i\right)}$
BLINEX	$\delta_{w}\left(\underline{x}\right)=\frac{-1}{q}*\text{Log}\left[we^{-q\delta_{0}\left(\underline{x}\right)}+\left(1-w\right)E\left(e^{-q\psi }|\underline{x}\right)\right]$	$\frac{-1}{q}\text{Log}\left[we^{-q\overset{\wedge }{\psi }}+\frac{1-w}{N-M}\overset{N}{\underset{i=M}{\sum }}e^{-q\psi^{\left(i\right)}}\right]$

**Table 2:** MSE of estimates for the parameter *a*.

(*n*, *m*)	Sc	MLE	Bootstrap		MCMC (*ω* = 0)			MCMC (*ω* = 0.6)		
			Boot-p	Boot-t	BSE	BLINEX		BSE	BLINEX	
						*q* = −0.5	*q* = 0.5		*q* = −0.5	*q* = 0.5
(30, 15)	I	0.0817	0.0953	0.0794	0.0773	0.0699	0.0613	0.0641	0.0652	0.0618
	II	0.0858	0.0864	0.0815	0.0836	0.0787	0.0629	0.0671	0.0743	0.0703
	III	0.0832	0.0814	0.0804	0.0842	0.0764	0.0645	0.0677	0.0781	0.0742

(30, 25)	I	0.0715	0.0919	0.0624	0.0579	0.0632	0.0508	0.0609	0.0733	0.5732
	II	0.0733	0.0971	0.0629	0.0592	0.0658	0.0513	0.0614	0.0751	0.0587
	III	0.0791	0.0957	0.0684	0.0588	0.0650	0.0521	0.0648	0.0769	0.0591

(50, 30)	I	0.0552	0.0647	0.0431	0.0418	0.0482	0.0322	0.0425	0.0498	0.0398
	II	0.0597	0.0654	0.0458	0.0432	0.0487	0.0348	0.0449	0.0509	0.0410
	III	0.0606	0.0662	0.0465	0.0444	0.0497	0.0384	0.0461	0.0527	0.0413

(70, 40)	I	0.0467	0.0614	0.0444	0.0356	0.0442	0.0314	0.0382	0.0492	0.0413
	II	0.0474	0.0619	0.0448	0.0383	0.0457	0.0327	0.0398	0.0515	0.0475
	III	0.0476	0.0632	0.0451	0.0386	0.0462	0.0356	0.0395	0.0467	0.0453

(80, 50)	I	0.0292	0.0325	0.0244	0.0124	0.0259	0.0119	0.0216	0.0235	0.0132
	II	0.0293	0.0331	0.0232	0.0135	0.0261	0.0127	0.0222	0.0254	0.0132
	III	0.0281	0.0279	0.0211	0.0127	0.0263	0.0131	0.0228	0.0252	0.0132

(100, 75)	I	0.0169	0.0214	0.0155	0.0098	0.0188	0.0097	0.0109	0.0125	0.0105
	II	0.0187	0.0229	0.0163	0.0129	0.0191	0.0098	0.0111	0.0140	0.0109
	III	0.0189	0.0287	0.0161	0.0113	0.0190	0.0098	0.0110	0.0139	0.0114

**Table 3:** MSE of estimates for the parameter *b*.

(*n*, *m*)	Sc	MLE	Bootstrap		MCMC (*ω* = 0)			MCMC (*ω* = 0.6)		
			Boot-p	Boot-t	BSE	BLINEX		BSE	BLINEX	
						*q* = −0.5	*q* = 0.5		*q* = −0.5	*q* = 0.5
(30, 15)	I	0.0643	0.0473	0.0198	0.0236	0.0277	0.0179	0.0275	0.0372	0.0259
	II	0.0653	0.0472	0.0205	0.0261	0.0283	0.0185	0.0285	0.0384	0.0254
	III	0.0931	0.0856	0.0228	0.0293	0.0286	0.0184	0.0289	0.0369	0.0267

(30, 25)	I	0.0480	0.0244	0.0172	0.0213	0.0234	0.0142	0.0276	0.0281	0.0162
	II	0.0591	0.0266	0.0175	0.0267	0.0253	0.0144	0.0289	0.0293	0.0275
	III	0.0485	0.0269	0.0242	0.0234	0.0273	0.0151	0.0295	0.0343	0.0279

(50, 30)	I	0.0400	0.0396	0.0158	0.0202	0.0251	0.0138	0.0239	0.0279	0.0261
	II	0.0518	0.0467	0.0127	0.0211	0.0298	0.0141	0.0240	0.0284	0.0269
	III	0.0793	0.0491	0.0174	0.0259	0.0273	0.0149	0.0245	0.0285	0.0298

(70, 40)	I	0.0391	0.0381	0.0123	0.0198	0.0212	0.0122	0.0205	0.0231	0.0198
	II	0.0435	0.0399	0.0199	0.0209	0.0238	0.0138	0.0217	0.0249	0.0215
	III	0.0669	0.0386	0.0162	0.0237	0.0242	0.0127	0.0233	0.0245	0.0219

(80, 50)	I	0.0352	0.0256	0.0198	0.0112	0.0131	0.0105	0.0129	0.0157	0.0117
	II	0.0372	0.0272	0.0185	0.0192	0.0135	0.0113	0.0138	0.0160	0.0130
	III	0.0464	0.0266	0.0166	0.0193	0.0133	0.0113	0.0142	0.0159	0.0130

(100, 75)	I	0.0133	0.0119	0.0079	0.0039	0.0055	0.0034	0.0098	0.0118	0.0064
	II	0.0136	0.0125	0.0095	0.0072	0.0084	0.0049	0.0098	0.0132	0.0076
	III	0.0139	0.0139	0.0116	0.0074	0.0098	0.0062	0.0104	0.0129	0.0097

**Table 4:** MSE of estimates for the parameter *α*.

(*n*, *m*)	Sc	MLE	Bootstrap		MCMC (*ω* = 0)			MCMC (*ω* = 0.6)		
			Boot-p	Boot-t	BSE	BLINEX		BSE	BLINEX	
						*q* = −0.5	*q* = 0.5		*q* = −0.5	*q* = 0.5
(30, 15)	I	0.0639	0.0588	0.0324	0.0381	0.0439	0.0353	0.0450	0.0464	0.0378
	II	0.0646	0.0639	0.0331	0.0410	0.0475	0.0404	0.0467	0.0492	0.0393
	III	0.0684	0.0628	0.0334	0.0439	0.0444	0.0417	0.0468	0.0496	0.0429

(30, 25)	I	0.0552	0.0653	0.0419	0.0358	0.0451	0.0349	0.0407	0.0415	0.0398
	II	0.0589	0.0524	0.0437	0.0395	0.0469	0.0354	0.0429	0.0416	0.0443
	III	0.0605	0.0639	0.0445	0.0388	0.0460	0.0351	0.0426	0.0427	0.0542

(50, 30)	I	0.0495	0.0447	0.0340	0.0309	0.0397	0.0295	0.0349	0.0364	0.0337
	II	0.0522	0.0491	0.0342	0.0324	0.0390	0.0348	0.0351	0.0397	0.0338
	III	0.0529	0.0490	0.0327	0.0398	0.0393	0.0366	0.0366	0.0397	0.0358

(70, 40)	I	0.0335	0.0294	0.0145	0.0261	0.0279	0.0175	0.0299	0.0230	0.0200
	II	0.0370	0.0378	0.0198	0.0297	0.0279	0.0178	0.0305	0.0247	0.0254
	III	0.0388	0.0355	0.0179	0.0319	0.0279	0.0178	0.0308	0.0242	0.0239

(80, 50)	I	0.0151	0.0149	0.0116	0.0181	0.0233	0.0113	0.0197	0.0221	0.0155
	II	0.0164	0.0149	0.0118	0.0116	0.0184	0.0101	0.0125	0.0171	0.0120
	III	0.0195	0.0173	0.0173	0.0226	0.0250	0.0135	0.0256	0.0231	0.0157

(100, 75)	I	0.0111	0.0103	0.0109	0.0108	0.0133	0.0094	0.0125	0.0152	0.0103
	II	0.0113	0.0120	0.0117	0.0109	0.0167	0.0099	0.0127	0.0165	0.0117
	III	0.0118	0.0108	0.0121	0.0116	0.0184	0.0101	0.0125	0.0171	0.0120

**Table 5:** MSE of estimates for the parameter *β*.

(*n*, *m*)	Sc	MLE	Bootstrap		MCMC (*ω* = 0)			MCMC (*ω* = 0.6)		
			Boot-p	Boot-t	BSE	BLINEX		BSE	BLINEX	
						*q* = −0.5	*q* = 0.5		*q* = −0.5	*q* = 0.5
(30, 15)	I	0.0302	0.0299	0.0248	0.0261	0.0279	0.0175	0.0299	0.0230	0.0200
	II	0.0397	0.0400	0.0249	0.0319	0.0279	0.0178	0.0308	0.0242	0.0239
	III	0.0371	0.0436	0.0258	0.0398	0.0393	0.0296	0.0366	0.0297	0.0358

(30, 25)	I	0.0233	0.0237	0.0199	0.0192	0.0135	0.0113	0.0138	0.0160	0.0130
	II	0.0324	0.0303	0.0219	0.0226	0.0250	0.0135	0.0256	0.0231	0.0157
	III	0.0347	0.0376	0.0289	0.0234	0.0273	0.0151	0.0295	0.0343	0.0279

(50, 30)	I	0.0262	0.0254	0.0246	0.0209	0.0238	0.0138	0.0217	0.0249	0.0215
	II	0.0286	0.0269	0.0249	0.0213	0.0234	0.0142	0.0276	0.0281	0.0262
	III	0.0291	0.0286	0.0254	0.0234	0.0273	0.0151	0.0295	0.0343	0.0279

(70, 40)	I	0.0178	0.0299	0.0147	0.0141	0.0169	0.0123	0.0142	0.0171	0.0143
	II	0.0203	0.0215	0.0153	0.0144	0.0174	0.0139	0.0151	0.0171	0.0149
	III	0.0218	0.0219	0.0198	0.0165	0.0183	0.0142	0.0159	0.0179	0.0157

(80, 50)	I	0.0163	0.0132	0.0164	0.0116	0.0134	0.0101	0.0125	0.0141	0.0120
	II	0.0165	0.0160	0.0155	0.0123	0.0139	0.0129	0.0143	0.0149	0.0146
	III	0.0166	0.0169	0.0147	0.0136	0.0154	0.0139	0.0145	0.0150	0.0150

(100, 75)	I	0.0098	0.0095	0.0093	0.0092	0.0105	0.0069	0.0096	0.0099	0.0073
	II	0.0106	0.0098	0.0094	0.0100	0.0114	0.0073	0.0103	0.0112	0.0098
	III	0.0111	0.0100	0.0096	0.0102	0.0115	0.0079	0.0100	0.0139	0.0098

**Table 6:** MSE of estimates for *r*(*t*) with *t* = 0.5.

(*n*, *m*)	Sc	MLE	Bootstrap		MCMC (*ω* = 0)			MCMC (*ω* = 0.6)		
			Boot-p	Boot-t	BSE	BLINEX		BSE	BLINEX	
						*q* = −0.5	*q* = 0.5		*q* = −0.5	*q* = 0.5
(30, 15)	I	0.0265	0.0254	0.0249	0.0237	0.0241	0.0225	0.0227	0.0230	0.0218
	II	0.0278	0.0271	0.0265	0.0251	0.0257	0.0238	0.0236	0.0235	0.0222
	III	0.0281	0.0283	0.0274	0.0259	0.0261	0.0241	0.0240	0.0239	0.0223

(30, 25)	I	0.0221	0.0199	0.0201	0.0185	0.0191	0.0192	0.0207	0.0216	0.0201
	II	0.0225	0.0219	0.0210	0.0187	0.0185	0.0196	0.0210	0.0223	0.0221
	III	0.0227	0.0221	0.0225	0.0191	0.0188	0.0198	0.0191	0.0219	0.0221

(50, 30)	I	0.0185	0.0175	0.0170	0.0125	0.0147	0.0121	0.0119	0.0098	0.0092
	II	0.0189	0.0183	0.0180	0.0134	0.0159	0.0125	0.0143	0.0141	0.0110
	III	0.0195	0.0193	0.0187	0.0149	0.0160	0.0129	0.0100	0.0115	0.0116

(70, 40)	I	0.0099	0.0100	0.0095	0.0088	0.0089	0.0090	0.0087	0.0088	0.0089
	II	0.0100	0.0113	0.0099	0.0089	0.0088	0.0087	0.0089	0.0089	0.0086
	III	0.0111	0.0115	0.0090	0.0085	0.0081	0.0083	0.0087	0.0088	0.0081

(80, 50)	I	0.0059	0.0054	0.0041	0.0029	0.0036	0.0021	0.0021	0.0025	0.0022
	II	0.0062	0.0059	0.0040	0.0034	0.0041	0.0030	0.0035	0.0032	0.0030
	III	0.0088	0.0073	0.0070	0.0072	0.0052	0.0061	0.0065	0.0050	0.0048

(100, 75)	I	0.0050	0.0049	0.0046	0.0031	0.0032	0.0037	0.0028	0.0033	0.0031
	II	0.0040	0.0045	0.0036	0.0021	0.0023	0.0033	0.0020	0.0025	0.0025
	III	0.0043	0.0041	0.0035	0.0025	0.0021	0.0022	0.0029	0.0030	0.0030

**Table 7:** MSE of estimates for *h*(*t*) with *t* = 0.5.

(*n*, *m*)	Sc	MLE	Bootstrap		MCMC (*ω* = 0)			MCMC (*ω* = 0.6)		
			Boot-p	Boot-t	BSE	BLINEX		BSE	BLINEX	
						*q* = −0.5	*q* = 0.5		*q* = −0.5	*q* = 0.5
(30, 15)	I	0.0100	0.0090	0.0099	0.0085	0.0085	0.0085	0.0093	0.0092	0.0093
	II	0.0100	0.0089	0.0099	0.0081	0.0081	0.0081	0.0089	0.0089	0.0089
	III	0.0100	0.0093	0.0099	0.0077	0.0077	0.0077	0.0085	0.0085	0.0085

(30, 25)	I	0.0100	0.0089	0.0100	0.0080	0.0080	0.0080	0.0089	0.0089	0.0089
	II	0.0100	0.0087	0.0100	0.0086	0.0086	0.0086	0.0092	0.0092	0.0092
	III	0.0100	0.0081	0.0099	0.0076	0.0076	0.0076	0.0085	0.0085	0.0085

(50, 30)	I	0.0100	0.0098	0.0100	0.0087	0.0087	0.0087	0.0093	0.0093	0.0093
	II	0.0100	0.0092	0.0100	0.0091	0.0091	0.0091	0.0095	0.0095	0.0095
	III	0.0100	0.0094	0.0100	0.0078	0.0078	0.0078	0.0087	0.0087	0.0087

(70, 40)	I	0.0100	0.0094	0.0100	0.0091	0.0091	0.0091	0.0095	0.0095	0.0096
	II	0.0100	0.0095	0.0100	0.0091	0.0091	0.0091	0.0095	0.0095	0.0096
	III	0.0100	0.0096	0.0100	0.0084	0.0084	0.0084	0.0087	0.0087	0.0087

(80, 50)	I	0.0100	0.0095	0.0100	0.0092	0.0092	0.0092	0.0096	0.0096	0.0096
	II	0.0100	0.0095	0.0100	0.0093	0.0093	0.0093	0.0096	0.0096	0.0096
	III	0.0100	0.0096	0.0100	0.0087	0.0087	0.0087	0.0090	0.0090	0.0091

(100, 75)	I	0.0100	0.0096	0.0100	0.0094	0.0094	0.0094	0.0097	0.0097	0.0097
	II	0.0100	0.0097	0.0100	0.0093	0.0093	0.0093	0.0095	0.0095	0.0095
	III	0.0100	0.0097	0.0100	0.0092	0.0092	0.0092	0.0094	0.0094	0.0094

**Table 8:** Point estimation for *a*, *b*, *α*, *β*, *r*(*t*), and *h*(*t*).

Method	*a*	*b*	*α*	*β*	*r*(*t*)	*h*(*t*)
MLE	0.1440	2.8097	0.3817	0.6267	0.9369	0.3397
Boot-p	0.2945	2.8094	0.9461	0.8919	0.9316	0.3647
Boot-t	0.2777	2.3717	0.6313	0.7247	0.9499	0.3267
MCMC	0.2846	2.4687	0.5223	0.6874	0.9305	0.3620

**Table 9:** 95% CI for *a*, *b*, *α*, *β*, *R*(*t*), and *h*(*t*).

Method	*a*	*b*	*α*
MLE	(-2.2774, 2.5654)	(-1.4917, 7.1111)	(-1.8837, 2.6471)
Boot-p	(0.0256, 7.1621)	(0.2122, 5.5427)	(0.0873, 7.9400)
Boot-t	(0.0164, 4.8129)	(0.2411, 5.7037)	(0.1326, 2.6246)
MCMC	(0.1265, 0.5103)	(1.6625, 3.4579)	(0.4884, 0.5876)
Method	*β*	*r*(*t*)	*h*(*t*)
MLE	(-0.7956, 2.0490)	(0.8651, 1.0088)	(0.0552, 0.6241)
Boot-p	(0.3261, 3.7536)	(0.7334, 1.0000)	(0.0004, 1.2423)
Boot-t	(0.4322, 5.6202)	(0.8248, 0.9999)	(0.0019, 1.0661)
MCMC	(0.6458, 0.7115)	(0.8370, 0.9823)	(0.1301, 0.6831)

**Table 10:** MCMC results for *a*, *b*, *α*, *β*, *r*(*t*), and *h*(*t*).

Parameter	Mean	Median	Mode	Variance	SD	ske
*a*	0.2846	0.2699	0.2510	0.0089	0.0944	0.8198
*b*	2.4687	2.4578	2.4212	0.2038	0.4514	0.2513
*α*	0.5223	0.5185	0.5108	0.0005	0.0220	1.2984
*β*	0.6874	0.6922	0.7020	0.0003	0.0176	-0.9618
*r*(*t*)	0.9305	0.9390	0.9527	0.0012	0.0351	-0.9926
*h*(*t*)	0.3620	0.3412	0.3144	0.0182	0.1350	0.6892

**Table 11:** Results of MLE and Bayes estimations.

Parameters	MLEs	*ω*	BSEL	BLINEX		
				*q* = −0.5	*q* = 0	*q* = 0.5
*a*	0.1440	0	0.2739	0.2871	0.2846	0.2821
		0.3	0.2387	0.2453	0.2424	0.2397
		0.6	0.1981	0.2025	0.2003	0.1981
		0.9	0.1576	0.1588	0.1581	0.1574

*b*	2.8097	0	2.4761	2.5198	2.4687	2.4196
		0.3	2.5762	2.6113	2.5710	2.5289
		0.6	2.6762	2.6987	2.6733	2.6444
		0.9	2.7763	2.7825	2.7756	2.7670

*α*	0.3817	0	0.5223	0.5225	0.5223	0.5222
		0.3	0.4801	0.4813	0.4801	0.4790
		0.6	0.4376	0.4392	0.4379	0.4367
		0.9	0.3957	0.3962	0.3957	0.3953

*β*	0.6267	0	0.6873	0.6875	0.6874	0.6873
		0.3	0.6691	0.6694	0.6692	0.6689
		0.6	0.6509	0.6512	0.6509	0.6507
		0.9	0.6327	0.6328	0.6327	0.6326

*r*(*t*)	0.9369	0	0.9321	0.9309	0.9305	0.9302
		0.3	0.9335	0.9327	0.9324	0.9322
		0.6	0.9350	0.9345	0.9344	0.9342
		0.9	0.9365	0.9363	0.9363	0.9363

*h*(*t*)	0.3397	0	0.3546	0.3671	0.3620	0.3570
		0.3	0.3501	0.3589	0.3553	0.3518
		0.6	0.3456	0.3507	0.3486	0.3466
		0.9	0.3411	0.3424	0.3419	0.3414

**Table 12:** Point estimation for *a*, *b*, *α*, *β*, *r*(*t*), and *h*(*t*).

Method	*a*	*b*	*α*	*β*	*r*(*t*)	*h*(*t*)
MLE	0.3254	2.5480	0.6245	1.3022	0.8038	0.3269
Boot-p	0.2583	2.8184	0.8306	1.5249	0.8616	0.3351
Boot-t	0.2284	2.7155	0.8721	1.5207	0.8603	0.3285
MCMC	0.2832	2.6328	0.7039	1.4972	0.8247	0.2904

**Table 13:** 95% CI for *a*, *b*, *α*, *β*, *r*(*t*), and *h*(*t*).

Technique	*a*	*b*	*α*
MLE	(-0.2527, 0.5514)	(1.2292, 3.8668)	(-0.3383, 1.5873)
Boot-p	(0.0780, 0.8932)	(0.9773, 3.1390)	(0.0834, 4.3518)
Boot-t	(0.0175, 0.9386)	(1.4634, 3.0890)	(0.2798, 3.3518)
MCMC	(0.0626, 0.5792)	(1.7626, 3.8057)	(0.3442, 1.0778)
Method	*β*	*r*(*t*)	*h*(*t*)
MLE	(-0.9338, 4.4720)	(0.6996, 0.9081)	(0.1457, 0.5081)
Boot-p	(0.4779, 4.5626)	(0.6503, 1.0684)	(0.1615, 0.4122)
Boot-t	(0.4755, 5.5563)	(0.6486, 0.9813)	(0.1764, 0.3533)
MCMC	(1.0544, 1.9124)	(0.7264, 0.9042)	(0.1876, 0.3934)

**Table 14:** Results obtained by MCMC technique for *a*, *b*, *α*, *β*, *r*(*t*), and *h*(*t*).

Parameter	Mean	Median	Mode	Variance	SD	ske
*a*	0.3325	0.3433	0.3342	0.0003	0.0164	0.0284
*b*	2.6328	2.6113	2.5589	0.2648	0.5146	0.4178
*α*	0.7039	0.7006	0.6940	0.0015	0.0394	0.3349
*β*	1.4972	1.2929	0.9652	0.0629	0.2508	0.8755
*r*(*t*)	0.8247	0.8243	0.8238	0.0021	0.0460	-0.3559
*h*(*t*)	0.2904	0.2872	0.2785	0.0035	0.0596	0.2811

**Table 15:** Results obtained by both MLE and Bayes MCMC estimation.

Parameter	MLEs	*ω*	BSEL	BLINEX		
				*q* = −0.5	*q* = 0	*q* = 0.5
*a*	0.3254	0	0.3267	0.3476	0.3325	0.3181
		0.3	0.3085	0.2975	0.2956	0.2955
		0.6	0.2094	0.2057	0.2007	0.2916
		0.9	0.1922	0.1922	0.1818	0.1741

*b*	2.5480	0	2.6375	2.7027	2.6328	2.5691
		0.3	2.5107	2.5684	2.5074	2.4561
		0.6	2.3839	2.4245	2.382	2.3491
		0.9	2.2571	2.2693	2.2566	2.2475

*α*	0.6245	0	0.7039	0.7043	0.7039	0.7035
		0.3	0.5853	0.5935	0.5853	0.5766
		0.6	0.4667	0.4763	0.4667	0.4573
		0.9	0.3481	0.3519	0.3481	0.3447

*β*	1.3022	0	1.5828	1.5951	1.5828	1.5826
		0.3	1.4082	1.4984	1.4983	1.4081
		0.6	1.3637	1.3739	1.3638	1.3635
		0.9	1.2291	1.2292	1.2291	1.2290

*r*(*t*)	0.8038	0	0.8245	0.8252	0.8247	0.8241
		0.3	0.6888	0.8236	0.8237	0.8233
		0.6	0.6969	0.8227	0.8228	0.8225
		0.9	0.7049	0.8218	0.8218	0.8217

*h*(*t*)	0.3269	0	0.2915	0.2913	0.2904	0.2896
		0.3	0.2966	0.2965	0.2959	0.2953
		0.6	0.3017	0.3017	0.3013	0.3010
		0.9	0.3069	0.3068	0.3068	0.3067

## Data Availability

The data set represents the survival times in years of a group of patients given chemotherapy and radiation treatment. For more details about these data sets, see Bekker et al. [20]. A generalization of the compound Rayleigh distribution: using a Bayesian method on cancer survival times. Communications in Statistics-Theory and Methods, 29(7), 1419-1433.
